This article has been retracted.

# The Influence Mechanism of BIM on Green Building Engineering Project Management under the Background of Big Data

**DOI:** 10.1155/2022/8227930

**Published:** 2022-10-10

**Authors:** Ning Feng

**Affiliations:** Henan University of Urban Construction, Pingdingshan 467036, China

## Abstract

The main framework of green construction management based on building information modeling (BIM) is constructed, and the related theories of BIM and green buildings are researched in more detail. The index of green construction is evaluated using the fuzzy evaluation method. The technical measures, management methods, field experience, and evaluation methods included in the green construction process are introduced in detail. Finally, effective measures to promote green construction management in China are proposed. This method is based on the specific technical measures and targeted management methods adopted in the green construction process. At the same time, the specific measures of construction project management in the era of big data are analyzed. It includes the collection and processing of data, the establishment of basic data models, the intelligent technology of big data clusters, and the application of blockchain big data. The purpose of the research is not only to effectively promote the development process of green construction in China, but also to reduce the waste of resources and environmental damage in the construction projects. At the same time, in the process of solving China's environmental protection, building construction must follow the guiding suggestions put forward under the green construction. This has an important reference value for promoting China's green construction work and has certain construction significance for realizing the sustainable development of the construction industry.

## 1. Introduction

According to the United Nations data, by 2030, China's urban population will reach the one billion mark. To satisfy the Chinese urban dream, China is bound to build large-scale urban living spaces and solve the resulting energy crisis. Correspondingly, China's construction industry will also face severe challenges. Such a large-scale new building with a huge amount of engineering not only faces strict cost control by the owner, but also faces the requirement of shortening the project cycle. On the other hand, with the continuous improvement of architectural aesthetic standards, architectural expressions are increasingly demanding freedom, unrestrainedness, and diversification [1, 2].The continuous emergence of special-shaped buildings and large-scale buildings has increased the difficulty of design and construction. Therefore, the future of China's construction industry will be more business, heavy workload, high efficiency, and low cost. It is also necessary to consider the modeling design and energy saving and environmental protection, and the difficulty of the challenge can be seen. In recent decades, productivity levels in the construction industry have not seen a fundamental increase globally. The root causes are the following two points [3, 4].One is because of the complexity and non-standardization of engineering projects. With the increase of construction participants, it brings great difficulties to the coordination among the participants. The synergistic effect between the participants also plays an increasingly important role in the success or failure of the project construction. The second is because it is difficult for all participants to obtain the massive data of the project in real time. The management process cannot be based on real-time accurate data, but can only rely on past experience. It is these two reasons that lead to serious delays, errors, and waste in engineering projects. But the current management techniques and methods cannot fundamentally solve these two aspects [5].

Building information modeling (BIM) technology [6, 7], as a general term for digital modeling software, parameterizes real building information in a virtual environment. Nowadays, to gain a leading edge from the fierce competition, enterprises need to use information technology to change the original situation of the construction industry that relies on a large amount of capital, technology, and labor input. BIM technology can allow information technology to form asset changes. The changed assets bring additional profits and form the core value of competition in the industry chain. This is also in line with the nature of informatization. The essence is to achieve high-quality control in a low-cost way. And it can realize information sharing and seamless docking. Therefore, the application level of BIM technology reflects the company's intensive management level to some extent. In-depth promotion of the development and construction of enterprise BIM technology is not only in line with the needs of the scientific development concept, but also the future development direction of the construction industry.

In recent years, the concept of BIM technology has not only been highly valued by academia and software developers, but the government has also issued some guidelines on BIM application. At present, BIM technology and BIM standards are gradually being researched commercially in China, and various application software applications are also being gradually explored and developed. At the same time, the research on construction project management based on BIM technology, as a breakthrough in the information management of the construction industry, is gradually being valued by various enterprises.

Figure 1 shows the change law of the total output value and the number of construction companies applying BIM in the construction industry in the past ten years.

The significance of this study is as follows:

In the face of increasingly fierce industry competition and deteriorating external environment, how to keep up with the development trend of the construction industry and establish a foothold in the industry is a key problem that every real estate development company needs to solve urgently. In view of the current social and economic development situation, BIM technology is becoming a new opportunity for the rapid development of construction engineering enterprises in the information age. It will fundamentally change the traditional management mode of green building engineering projects, and also bring advanced technology and new blood to green building engineering enterprises. The application research of BIM technology has also received extensive attention from academia and business circles. Therefore, the research on the application of BIM technology to green building project management has the following significance [8, 9].

(1) This study starts from the perspective of how to improve the core competitiveness of construction engineering enterprises. Combined with the development status and background of domestic and foreign BIM technology and the development and application practice of BIM technology in China's green building engineering projects, the research on the impact of BIM technology on engineering project management is carried out. This is the enrichment and expansion of the application methods and research in the field of construction project management in China, and has important theoretical value.

(2) This article studies the development achievements of BIM at home and abroad, mainly studies the practice of BIM technology in the management of green building engineering projects. The research on the application process of BIM technology will have an important practical guiding significance for the improvement of engineering project management design quality, production efficiency, and competitiveness of construction engineering enterprises.

In a word, this research topic selected in this study has very important theoretical and practical significance for both the theoretical promotion of BIM and its practical application in green building project management.

## 2. Theoretical Overview of BIM Technology

### 2.1. The Concept of BIM Technology

BIM focuses on recording the data of the entire life cycle of engineering buildings, which is a dynamic process. Compared with traditional 3D drawing, BIM adds the concept of time. In the beginning, the basic definition of BIM is not perfect. There are four main stages of evolution in the name BIM. The most basic simple 3D modeling is a digital building, a mid-term virtual building, a mid-late building product model, and a professional building information and model for the entire life cycle of the building that can be generated in the later stage [10, 11].Therefore, BIM is ultimately defined as a kind of building information and model. It has gradually become a specialized and technical term widely recognized in the construction industry. The basic concept of BIM originally came from the famous American Professor Charlie Eastman. He once thought that the information model of a building is the geometric information of all the sizes and dimensions of a building or structure in the whole life cycle of its project. At the same time, it integrates non-geometric information during construction into a building model.

With the continuous in-depth promotion and innovation of BIM technology in practice, many institutions and users engaged in BIM research have different concepts and interpretations of BIM technology. However, because China's BIM standard started relatively late in practice and application, it is still in its trial period, and there are various disputes over its definition. Therefore, this study basically adopts the definition of foreign BIM standards, and the specific content can be divided into three aspects [12].

(1) Construction projects can use BIM technology to build their models. The various physical data information and functional properties of construction projects are added to the model. The international standard BIM requires specific architectural engineering models to be digitally expressed.

(2) It is necessary to integrate the BIM models in the same engineering platform into the professional construction information and data of the entire engineering project. It acts as a shared information and data resource. The data in the whole life cycle of conceptual design, preliminary planning, construction map design, construction, operation management, and maintenance of the same project can be described through the level of detail of BIM model information in different periods of the same platform. It also provides engineering decision-making basis for decision-makers.

(3) The platform based on BIM technology in different development stages of the construction project, the participants of the construction project have the right to authorize the authority based on the BIM-based platform. Through the BIM model, the project data within the authority is automatically extracted, applied, and updated to cooperate with the participants of the construction project.

### 2.2. The History of BIM

Since the founding of New China, the rapid development of industrialization has provided a huge impetus to the national economy, and various industries in the industrial system have also made leap-forward progress. Compared with other traditional industries, such as the textile industry, electric power industry, and automobile manufacturing industry, the development of construction industry is relatively lagging. Therefore, the market demand for the improvement and transformation of the construction industry is more and more urgent [13]. After analyzing and comparing the development history of other industries, it is found that the improvement path is mainly the application of new technologies and new management models. The application of the two is gradually developed and expanded based on the information platform. Therefore, to improve the quality and efficiency of the construction industry, the key point is “informatization.”

Looking back at the development of construction industry informatization, it can be divided into three stages.

(1) The appearance of computer aided engineering (CAE) changed the calculation problem in engineering design from manual operation to computer-aided operation.

(2) CAD drawing software makes computer drawing replace manual drawing, which greatly improves work efficiency.

(3) The emergence of BIM provides technical support for the construction industry to enter the deepening stage of informatization. It also realizes the transformation of information from two-dimensional drawings into three-dimensional models.

The current construction industry informatization can be divided into two parts: technical informatization and management informatization. The main applications are shown in Figure 2.

As can be seen from Figure 2, in the construction industry informatization, the vertical information flow is basically opened up. However, there is a lack of connection between horizontal information, and they are still in a state of independent work. From a macro perspective, there are barriers between technology informatization and management informatization, and they go their separate ways. From a microscopic point of view, there is a lack of connectivity among various disciplines [14].

It is analyzed from two aspects of technology informatization and management informatization. Technology informatization should cover the entire life cycle of buildings. However, in the whole life cycle, the informatization in the construction stage is often weakened or even ignored, and the focus is more on the pre-planning and design stages. The core goal of management informatization is to effectively manage enterprise resources. No matter what kind of informatization it is, the main body it faces is the construction project itself. Therefore, the key to realizing the informatization of the construction industry lies in the effective integration and application of information. The core value of BIM technology is informatization, including the integration and analysis of building information. It can integrate the information required in the construction process into a model to realize information sharing and mutual guidance. Thereby, the barriers between technology and management and between various professions can be broken. It can become the link of horizontal connection of information.

### 2.3. Advantages of BIM Technology in Green Construction Information Management

The application of BIM technology to the green construction informatization management process is a transformative leap in the informatization process of the traditional construction industry. Several advantages of BIM technology can just make up for the problems and deficiencies in the current green construction informatization process [15].

#### 2.3.1. Visualization

The basis of using BIM technology is the establishment of an information model, and the whole process of construction is displayed by establishing a three-dimensional model of the building. It is quite different from the information management of traditional construction in the expression of information. In the traditional construction process, the understanding of buildings is based on complicated CAD drawings. The designer should divide the building into three perspectives: flat, vertical, and sectional. The construction personnel also need to construct a spatial image in their minds according to the two-dimensional drawings, and then carry out the construction. For some more complex projects or special-shaped buildings, it increases the difficulty of design and construction. BIM technology breaks through the previous thinking mode. It directly constructs a three-dimensional architectural model and expresses geometric information vividly. The corresponding viewing angle can be selected for observation according to the needs, which provides great convenience for the staff. The 3D building model makes the model intuitively understandable even for those who do not have a professional background. It is conducive to the communication, discussion, and decision-making of all parties involved in the project, thereby breaking the barriers of horizontal information exchange. The changes brought by BIM to engineering construction are shown in Figure 3.

#### 2.3.2. Integration

The high integration of information is another advantageous feature of BIM. The construction process is a complex, expensive, and time-consuming system engineering. In CAD drawings, the geometric information and physical properties of buildings and components are separated. To obtain the physical properties of a component, it is necessary to search according to the drawing index, which is very inefficient. In BIM technology, the model integrates the geometric data information of the building and the physical properties of the components. All information is displayed when viewing component properties, improving work efficiency. In addition, the relative independence of various types of information (architecture, electromechanical, progress, finance, etc.) results in engineering personnel of different majors only working for their own major. The lack of information exchange caused many problems in the actual construction. The multi-purpose function of BIM can integrate the results of different disciplines into the model. It provides a platform for breaking the barriers of information transmission and realizing professional collaboration. It also provides a basis for information sharing in the whole life cycle of buildings.

#### 2.3.3. Relevance

The relevance of BIM refers to the relevance of the same information in different dimensions, which can be summarized by “change all at once.” The construction process involves multiple disciplines, and how to ensure the timeliness and accuracy of information updates is one of the current difficulties. In the traditional construction process, a lot of time and energy are consumed in the modification of drawings. Once a change is required, professionals need to find the component in all the involved drawings and modify it one by one. Coupled with the lack of smooth communication channels between disciplines, lags, or errors are inevitable when changes are passed on to other professionals. The implementation of BIM treats each component as a unit. Any modifications made on it are reflected directly in the model. All parties involved in the project can receive and provide feedback in a timely manner. The integrity and timeliness of the information is guaranteed.

#### 2.3.4. Simulation

If the changes brought by BIM to the construction industry are summarized as “two-dimensional to three-dimensional,” then this perspective changes. The replacement process also provides a new idea of construction management and control on the basis of the three-dimensional model. In traditional construction, multi-disciplinary projects need to be carried out at the same time most of the time. It is difficult for an engineering personnel to predict the problems encountered during the construction of the building. Simple building outline frame is far from meeting the needs of practical engineering. BIM can link schedule and cost documents on top of the 3D models. Through a series of settings, it can be observed whether the changes in the construction progress and cost of the building information model meet expectations as the construction progresses. In this way, construction simulation can be carried out from different professional perspectives, and construction simulation can be carried out directly on the integrated model to achieve the purpose of precise control.

#### 2.3.5. Optimization

The construction project from pre-planning, design, and construction to operation and maintenance is actually a process of continuous optimization, adjustment, and continuous improvement. Based on the above four advantages of BIM technology, it can be seen that the building information model has the integrity and accuracy of information. At the same time, there are powerful real-time update and simulation functions, which provide a guarantee for the optimization of construction plans. A building information model integrates all geometric and physical characteristic data of a building. It enables multi-professionals to perform collision checking in the model to find errors. At the same time, the model can correlate progress and cost documents, and simulate after combining the objectives of quality, cost, progress, and environmental protection. It is required for optimization based on the results calculated by different schemes. It not only improves the scientificity and effectiveness of decision-making, but also helps to reduce costs and shorten the construction period.

### 2.4. Features of BIM Technology

3D visualization breaks through the limitations of 2D CAD drawing. The model can be used to display the actual situation of the building structure, which can replace the traditional projection method of 2D drawings to represent the building entity. It can directly and completely display the building in three dimensions. Thereby, it can truly imitate the real object of the building and reflect the application value of the technology [16, 17].

In project design, collaborative design breaks through the connection between the upstream and downstream of traditional majors and solves the limitations that majors cannot collaborate and information cannot be shared in time. The focus is on solving the problem of non-coordinated design between disciplines. The platform built by BIM technology solves the problems that arise during the design. It is necessary to provide an instant and effective communication design platform for the project operation and design process, which can record complete architectural design information data.

The optimized construction scheme is mainly reflected in the individualized design for the schemes that are difficult to construct and have many construction problems during construction. Through the construction simulation process of the BIM 3D model, the deepening of the optimization tools can be matched. The general optimization content can be completed in the early stage of construction. Therefore, most projects can effectively reduce project risks and save project costs after optimization.

Drawing a 3D model through BIM technology not only improves the accuracy of the 2D drawings of complex buildings, but also can be applied to drawing optimization and personalized drawing customization. It can show the practical application value of the simulability and optimizability of drawings more.

## 3. Influence Analysis of BIM Technology on Green Building Engineering Project Management

This chapter focuses on analyzing the impact of BIM technology on various management links in the life cycle of construction projects. The regularity of BIM technology in construction project management is extracted from it [18].

### 3.1. The Whole Life Cycle Management Mode of BIM Technology

#### 3.1.1. Design Unit-Led Model

In this management mode, design units can fully express their design intentions and ideas by using BIM technology. Especially for those large and complex construction projects, the design institute will apply BIM technology in advance to carry out the 3D design of engineering projects and make project BIM information models. The design concept needs to be presented to the image of the owner. It is necessary to effectively communicate with the owner through the BIM information system to strengthen the collaborative management of design projects.

#### 3.1.2. Construction Unit Leading Mode

The construction unit-led model means that the construction unit uses BIM technology to model and analyze the key and difficult points of the project before the project is implemented. By formulating a reasonable construction plan and using appropriate construction methods, the difficulties of the project can be effectively solved. Using BIM technology to guide construction can effectively improve the core competitiveness of construction companies and save operating costs. For the construction unit, since the BIM model contains information, such as the construction period and cost of the construction project, the BIM model can be extended from the three-dimensional management of the project management to the four-dimensional management. The construction progress and materials and equipment can be predicted, and the construction cost can be reasonably controlled. The four-dimensional construction simulation of BIM technology can vividly reflect the characteristics of the engineering structure. It can make the general contractor and other construction participants have a clear understanding of the project. At the same time, it can also combine the BIM information model to formulate appropriate construction plans and reasonably allocate labor. The optimization of engineering construction can be achieved within a given construction period.

#### 3.1.3. Owner-Unit-Led Model

The owner-dominant mode of BIM technology is gradually generated with the continuous development of BIM technology and the improvement of construction project management's demand for owner management. This BIM management model is a qualitative progress in the development of BIM technology. BIM technology has been recognized and promoted by the owner unit, and it is the most in line with the BIM development concept. The need to be led by the owner can promote the promotion and application of BIM technology in the whole life cycle of the construction project, and promote the efficient management of the project. The dominant mode of the owner unit greatly enhances the owner unit's control over the construction project and strengthens the management precision and management depth of the owner unit. It not only makes up for the shortcomings of individual owners' lack of engineering expertise and weak engineering management technical strength, but also provides a platform for collaborative communication between all participating parties in the construction project.

### 3.2. Research on the Application of BIM Technology in All Stages of the Whole Life Cycle

#### 3.2.1. Application Research of BIM Technology in Design Stage

The ultimate goal of implementing BIM technology in the design phase of architectural projects is to improve the quality and efficiency of project design. This will reduce engineering rework, waste of engineering materials, and delays in construction due to problems with design drawings in subsequent construction stages. Therefore, the construction period of the project can be reliably guaranteed and the project cost can be saved. The value of BIM technology in the design stage of architectural engineering is mainly reflected in the following aspects.

*(1) Visualization Performance of Construction Projects*. BIM technology can express professional and abstract two-dimensional building plans in the form of three-dimensional models. It has the characteristics of popular and intuitive. It enables all parties involved in the construction project to understand the project status simply and clearly. This in turn makes clear and efficient decisions for project implementation.

*(2) Promoting Collaboration among Various Disciplines*. BIM technology integrates the design content results of different disciplines, members, and systems of construction engineering in a unified 3D collaborative design environment. It avoids unnecessary design errors caused by different design ideas or untimely communication among design members of various majors, and improves design quality and efficiency.

*(3) Optimizing the Structural Characteristics of Construction Projects*. The above two features enable design optimization to be implemented smoothly. It ensures concise and efficient design results. This feature is especially important in complex architectural designs.

*(4) Drawability of Design Drawings*. Construction drawings based on BIM technology can be effectively displayed in floor plans. It guarantees the implementability of BIM technology implementation.

At the same time, the collaborative operation of BIM technology in the design stage is also reflected in the collaborative management of various design documents, office documents, permissions, design review, design plans, and project status query statistics other than design drawings. At the same time, BIM technology is also a collaborative management platform for the design party and the owners, construction parties, supervisors, material suppliers, operators, and other project participants to exchange documents and communicate with each other. It is an important means to improve the management efficiency of each stage of the project management life cycle.

#### 3.2.2. Research on the Application of BIM Technology in the Construction Stage

The application of BIM technology in the construction stage is mainly reflected in the following aspects.

(1) Through 3D simulation modeling, the publicity results of the project can be improved. By simulating the construction project in 3D, the simulation model can give people a strong sense of reality and direct visual sense.

(2) Through the BIM information integration capability, rapid calculation and efficiency improvement can be achieved. Through the establishment of the BIM database of construction projects, a project-related database can be established. The required engineering quantity can be calculated accurately and quickly in the database. It greatly improves the accuracy and efficiency of the construction budget, and can quickly extract the project data information required by the project management process and nodes. This effectively improves the efficiency of project management.

(3) It can effectively avoid waste. The refined management of construction enterprises is often difficult to achieve. The fundamental reason is that construction engineering has huge engineering data. It makes the traditional project management method unable to obtain the required resources quickly and accurately. All project management relies on construction experience, which will inevitably lead to waste of resources and delay of construction period.

(4) Through the model, the construction process can be virtualized and the effective coordination of project management can be promoted.

(5) Through BIM modeling, piping, and structural collision checking can be performed and rework during construction can be reduced.

(6) BIM model can call and synthesize all relevant data of construction engineering, and provide decision support for engineering decision makers. The engineering data in the BIM data model have the characteristics of fusion and quantification. BIM database provides a large amount of engineering information for engineering. These basic data can be coordinated and shared among the participating construction management departments. All engineering quantity information can be aggregated and split according to time and type for comparative analysis. These characteristics of the BIM model ensure that the basic engineering data are provided to the required construction parties in a timely manner. It provides an important basis for project decision makers to participate in project management and make project decisions.

## 4. Analysis of the Development of BIM in China's Construction Projects

### 4.1. Current Situation of Construction Project Management in China

In the course of more than 30 years of development, China's project management has achieved remarkable results. However, problems such as quality accidents, delays in construction schedules, and budget overruns are not uncommon. Especially in recent years, there have been many accidents involving the breach of the Jiujiang Yangtze River dyke, the serious accident of the Ningbo Bridge, and the quality problems of the Beijing West Railway Station. While causing huge losses to the life and property of the country and the people, it also sounded the alarm for the current situation of China's construction project management. Poor management and non-standard management are the main reasons for these accidents. This shows that there is still a huge gap between China's construction project management level and foreign developed countries, and there are still many problems to be solved urgently.

Figure 4 shows the proportion of major accidents caused by construction project management level in the past ten years.

It can be seen from Figure 4 that the proportion of accidents caused by non-standard management methods is the largest, and the proportion of accidents caused by design changes is the smallest. Project management models and controllable design requirements also need attention. Although the proportion of the two ranks at the bottom, but the proportion of both exceeds 20%.

### 4.2. The Shortcomings of Traditional Construction Project Management

The deficiencies are described in detail as follows.

#### 4.2.1. Phase Fragmentation in the Project Life Cycle

The whole life cycle of a typical construction project includes project decision-making and preliminary preparation stage, project implementation stage, and project operation stage. There are intrinsic links between activities throughout the life cycle. The output of the previous stage project is the input of the subsequent stage project. When carrying out a certain stage of work, due to different implementation subjects, insufficient information communication, or self-interested motives of the implementers, it may be difficult for the activities of this stage of the project to fully absorb the work results of the previous stage. Implementers also rarely consider the impact on later stages of work. For example, in the design stage, designers mainly design according to the design requirements put forward by the construction unit and relevant national design regulations. They rarely regard construction convenience as an external constraint, and sometimes even design solutions that are extremely difficult to construct.

#### 4.2.2. There Is a Large Conflict of Interest among the Project Participants and the Various Departments of the Team

For the same project, each participant tends to prioritize the goals according to their own responsibilities in achieving the goals. They will prioritize goals within their primary responsibilities, and make coordinating goals with others a secondary goal. Due to the inconsistency of goals, there is a check-and-balance phenomenon among the project participants, which leads to tension in the organizational relationship and low work efficiency. At the same time, the enthusiasm and creativity of all parties are inhibited, and a lot of cost, time and energy are also consumed in the coordination of various work interfaces. For example, there is a conflict of interest between the owner and the contractor of a construction project. Under the premise of satisfying the function, quality and progress, the owner pursues the smaller investment, the better. This is in fundamental conflict with the contractor's pursuit of profit maximization.

#### 4.2.3. There Is a Serious Division between the Majors of the Project

During the design process, there is a phenomenon of “fighting” among the five major designers of architecture, structure, water supply and drainage, HVAC, and strong and weak electricity due to poor communication. In the construction process, especially in the installation stage, there are intricate inherent constraints and connections between the four major professional processes. There are many sub-contractors involved, and there is often a phenomenon that the work interface is not coordinated. Especially in the case of tight construction schedules, it is easy for them to fight each other regardless of the internal connection between the processes in order to complete their respective schedules. This results in cross-contamination or even destruction of the finished product.

#### 4.2.4. Poor Information Exchange and Communication among the Participants

A large construction project usually involves hundreds or thousands of participants to complete thousands of procedures or activities. The smooth implementation of each process or activity relies on a large amount of information. Therefore, the acquisition, storage, analysis, and processing of information and the effective communication among the participants play a crucial role in the realization of the project objectives, and are the key to the success of a project. For large-scale construction projects, the complexity of the large number of participants, processes, and activities increases the amount of information. At the same time, it also increases the difficulty and importance of information management.

### 4.3. Analysis on the Limiting Factors of Green Building Project Implementation

Construction projects have a long construction period and a large amount of work. Factors, such as the professionalism of the project and the number of participants lead to the obstruction of corresponding information during the implementation of the project. The same green building project has more participants and more professional parties than traditional building projects. At the same time, the difficulty of evaluating green building standards in the process of green building is also a factor limiting the implementation of green building projects [19–21].

#### 4.3.1. Inefficient Information Transfer between Various Stages of the Project

From the perspective of the whole process of green building project implementation, the biggest challenge in green building project implementation process is poor information dissemination. The specific performance is as follows.

*(1) Building Information Is Complex and Difficult to Store*. The information storage of green building projects is mainly divided into two categories. The first category is structured information. It refers to the information stored in the CAD drawings, such as the floor plans of various professional buildings, the length, width and height of building components, and the corresponding building materials. The second largest category is non-fully structured building structure information. Such structural information includes contracts, photos, or videos on the project. For green buildings, it is difficult to store building information in the same building information model. In the past ten years, the proportion of structured and unstructured building information to green building information is shown in Figure 5. At present, it is the structural building information that is convenient to communicate and manage in the process of information management. Most of the non-structural ones that are not suitable for sharing, storage, and management seriously hinder the transmission of green building information and the implementation of green building projects.

*(2) Repeatability of Information Transfer between Phases of Green Building Projects*. Green building project management is full life cycle project management. In different stages of project implementation, each major needs to do a good job of professional information transmission. Since the majors of the project participants at different stages of the project are different, the information that different majors and different participants of the project pay attention to in the process of project transmission are different. This not only leads to a vicious circle of building information being created, lost, re-established, and lost again, but also a fault in building information.

#### 4.3.2. Poor Coordination of Various Disciplines during the Implementation of the Project

Compared with traditional project management, green building project management involves more project participants. At the same time, the requirements for multiple building materials and design are higher, and the various participants of the project in the process of green building implementation (as shown in Figure 6). In the green building implementation project, the professional requirements are very high. However, the degree of cooperation between different majors is relatively low. In the process of project design, construction, operation, and maintenance, the problem of collaborative work is more prominent.

### 4.4. Demand Analysis of the Development of BIM in Construction Projects

The rapid development of computer software and hardware as well as high-tech has provided a source of power for the development of BIM. The information platform for collaborative management will become more and more convenient and standardized. Even the physical model can be directly generated by 3D printer, these are the future development directions of BIM.

(1) In the current development process of the construction industry, there is a shortage of BIM technical talents. In the process of project management using BIM technology, the management of talents is also very important. Therefore, training BIM technical talents and management talents has become a top priority on the road of BIM development. As a developer of a construction project, there should be a BIM manager at the same level as the manager in charge of the project. They are responsible for the development, operation, and maintenance of BIM projects and have the authority to edit any information in the building information model at will. The BIM manager should first have the ability to control and understand 3D BIM software. They not only have rich experience in BIM projects but also have leadership skills in the development, maintenance, and team building of BIM models. In the early stage of a construction project, it is necessary to rely on the BIM experience of the BIM manager to avoid BIM problems that may be encountered later. This can make the demonstration phase of the project more detailed and reliable.

(2) There should also be a BIM Supervisor in the BIM team. The person is responsible for analyzing and summarizing various professional information in the BIM model and reporting it to the BIM manager for decision-making. BIM supervisors should be familiar with various operational processes of BIM project management and proficient in various tools for operating BIM. This facilitates resource sharing and information sharing among various disciplines.

(3) BIM projects should also have professional managers. In the pre-design process of the project, it is inseparable from the coordination and communication of professional managers who are familiar with BIM software and have a high level of professional ability. The workload at this stage is very large, which is much more complicated and more difficult than the two-dimensional drawing design. In the construction project of BIM application, each professional manager is the direct operator and provider of BIM model information. Therefore, the quality of the project depends on their BIM operation ability and experience, as well as their professional ability and management ability.

### 4.5. Advantages of Project Management Based on BIM Technology

The BIM-based project management model is to create, manage, and share information in a digital way. It has many advantages:

(1) The ideal control of capital risks and profit goals in a short period and in the whole process can be fully realized.

(2) Based on BIM technology, budgets, tenders, progress audits, and settlements can be managed in a unified manner, and data comparison can be formed.

(3) It can manage the cost of the whole process of cost budget, bidding, visa management, fee payment, and so on. It can also provide construction contracts, payment vouchers, construction changes, and other project attachment management.

(4) The BIM data model ensures that the data of each project are dynamically adjusted. It is convenient to count and trace the cash flow and capital status of each project.

(5) BIM-based 4D virtual construction technology can detect problems that may arise during the construction phase in advance. Before construction starts, one by one modification, corresponding countermeasures can be formulated.

(6) The introduction of BIM technology can fully exploit the potential energy of traditional technology. It can make it more fully and effectively serve the quality management of engineering projects.

The use of BIM technology enables the entire engineering project to effectively establish resource plans, control capital risks, save energy, save costs, reduce pollution, and improve efficiency in the stages of design, construction, operation, and maintenance. The application of BIM technology can not only change the traditional project management concept, but also lead the building information technology to a higher level. Thereby, the integration degree of building management can be greatly improved.

## 5. Specific Measures for Construction Project Management in the Era of Big Data

In the era of big data, there are strict requirements for the management of construction projects. In the implementation, it needs to be clearly managed to ensure the overall feasibility. The specific measures are analyzed below [22].

### 5.1. Collection and Processing of Data

In the process of project construction, a large amount of data may be generated, which requires efficient management by managers. In the data collection stage, there are many types of actual construction project management. For construction projects, in the process of using big data technology to collect and organize, managers need to do a good job in data collection, data storage, and integrated analysis. Master the project trends of future construction projects and strengthen the research and application of virtual community data technology. In addition, in the process of applying big data information technology, managers will implement big data technology and target planning and target control of construction projects. It is necessary to ensure the authenticity and reliability of data content in the process of deepening big data technology. Finally, engineering managers should pay attention to data management and requirements in the big data application stage. It is necessary to connect it with other engineering projects, and deepen the technological innovation on the existing basis, so as to achieve the desired results.

### 5.2. Establishment of a Basic Data Model

In the data analysis of construction projects, according to the requirements of big data, it is necessary to actively construct the basic data model to help project managers obtain scientific management methods. Under the basic data model, construction project management needs to fully grasp the corresponding data and information. Integrate various data by exploring the rules and content. By focusing on the management process of data information, the actual connection is realized. In operation, the general characteristics of construction projects are displayed with the help of basic digital and analog models. In view of the phenomenon of non-standard construction in the construction stage, the relevant personnel must clarify the specific module content. If the control is not in place, the coefficient should be adjusted to ensure the controllability of the project.

### 5.3. Big Data Cluster Intelligence Technology

Intelligent analysis and application can be carried out in the process of current innovation management. Managers are required to be good at adopting intelligent management techniques. It is necessary to realize the digital management of construction projects across time and space in integrated analysis. Starting from planning and design, construction management and operation, we will provide multiple supply chains in future intelligent buildings, and then realize integrated assembly management. It needs to be coordinated in the follow-up management. Modern technologies are used in construction site management and control, including large-scale data collection and analysis technology represented by drones, and RFID technology. Ultimately, the overall rationalized management is realized.

### 5.4. The Application of Blockchain Big Data

In the current context of big data, the technical form of blockchain big data is highly feasible. This type of technical form mainly refers to the technical form of security application for the network transmission form of data information. Encryption algorithms, point-to-point transmission, and distributed data storage are involved in the whole stage. In the application of various information technologies, managers need to reasonably apply the form of big data in the blockchain. The complete model framework constructed is shown in Figure 7.

To sum up, in the context of the era of big data, the management of construction projects should pay attention to its rationality. This study comprehensively analyzes the contents of project management and the treatment of corresponding problems, so as to ensure the safety of engineering projects and achieve overall development.

## 6. Evaluation Index System of the Impact Mechanism of Green Building Project Management Based on BIM

### 6.1. Principles of Establishing an Evaluation System

The evaluation system is the basis for evaluation. The evaluation index of the impact mechanism of BIM on green building project management is based on the content of green building project management. The following principles should be followed during the establishment process [23, 24].

#### 6.1.1. Comprehensiveness of Indicators

When the indicators are determined, it is necessary to comprehensively determine the indicators of the impact mechanism of BIM on green building project management and ensure sufficient coverage. At the same time, the indicators at all levels of its impact mechanism are also required to be comprehensively covered.

#### 6.1.2. The Scientific Nature of the Indicators

In the process of evaluation, the establishment of the evaluation system is based on the content of green building project management. Therefore, the way in which the application of BIM technology affects it must be correct and scientific.

#### 6.1.3. Comparability and Operability

In the BIM analysis of the influencing factors of the green building project mechanism, the selected indicators should be representative and concise on the basis of satisfying the coverage. Metric requirements can be quantified. There are comparable conditions in the study of the impact mechanism of BIM on green building project management.

#### 6.1.4. Simplicity

The impact of BIM on green building project management is evaluated on the basis of BIM technology. Impact metrics need to be as simple and focused as possible. This can improve the success and accuracy of the evaluation.

### 6.2. Construction of Evaluation System

The evaluation index system is divided into two categories, including 5 first-level indicators and 17 second-level indicators. The second-level indicators have clear meanings and directly reflect the on-site “green” performance of the construction companies. The specific meaning of the first-level and second-level indicators is explained below.

#### 6.2.1. First-Level Indicators

*a* stands for section and land use protection. *b* stands for energy saving and energy utilization. *c* stands for material saving and material resource utilization. *d* stands for water saving and water resource utilization. *e* stands for environmental protection.

#### 6.2.2. Second-Level Indicators

*a*1 represents the temporary land for construction site. *a*2 represents the temporary land use area. *b*1 represents the quota measurement of construction energy consumption. *b*2 represents the full-load operation factor of the construction equipment. *b*3 represents new energy-saving technologies and new processes. *b*4 represents the energy use structure. *c*1 represents the use of recycled materials. *c*2 stands for in situ sampling. *c*3 represents the use of green building materials. *c*4 represents the use of industrialized products. *c*5 represents the material consumption quota measure. *d*1 represents water-saving processes, equipment, and facilities. *d*2 represents the quota measurement of construction water. *e*1 represents the construction area separation. *e*2 stands for environmentally friendly mechanical use. *e*3 represents the classified treatment and recycling of construction waste. *e*4 stands for ecological restoration.

### 6.3. The Weight of the Indicator Is Determined

The most commonly used analytic hierarchy process is used to determine the weight ratio of each evaluation index of green construction. This study is divided into three steps to calculate the weight [25].

#### 6.3.1. Construct Green Construction Evaluation Index Importance Degree Matrix

The first-level indicators are used as indicators and the second-level indicators are used as factors. For the evaluation index levels with the same degree of importance, the relative importance of each index is obtained by comparing the two, and the importance degree matrix *A* is formed as follows.

(1) $$\begin{array}{c} A=\left[\begin{array}{ccccc} Ck & A_{1} & A_{2} & \cdots & A_{n}\\ A_{1} & a_{11} & a_{12} & \cdots & a_{1n}\\ A_{2} & a_{21} & a_{22} & \cdots & a_{2n}\\ \cdots & \cdots & \cdots & \cdots & \cdots \\ A_{n} & a_{n1} & a_{n2} & \cdots & a_{nn} \end{array}\right]. \end{array}$$

According to the methods of empirical analysis and expert investigation, the elements *a_ij_* in the matrix are reflected in the same dimension using the 9-dimensional scaling method. *A_i_* and *A_j_* represent the importance of the associated meaning between elements. The relative importance of the analysis elements is scaled from 1 to 9 into 9 dimensions.

#### 6.3.2. Single Ranking and Consistency Analysis of Each Evaluation Index Level of Green Construction

The level of a single order in the hierarchical factors according to the evaluation system of each response factor has been selected. According to the basic principle of AHP, determine the maximum eigenvalue corresponding to the eigenvector of the matrix. The ability of factor ranking weights to be the relative importance of the target factor. After judging the matrix, it is a very important and critical link to carry out the necessary matrix consistency test to determine whether the weight of each index is contradictory.

*(1) Calculate the Largest Eigenroot of the Judgment Matrix*.

(2) $$\begin{array}{c} \lambda_{\max}=\frac{1}{n}\overset{n}{\underset{i=1}{\sum }}\frac{{\left(AW\right)}_{i}}{W_{i}}, \end{array}$$

where *A* represents the entire judgment matrix. *W* represents the eigenvectors of the judgment matrix. AW*_i_* represents the value of the *i*th element of the vector AW.

*(2) Calculate Consistency Metrics*.

(3) $$\begin{array}{c} \text{CI}=\frac{\left(\lambda_{\max}-n\right)}{n-1}. \end{array}$$

When the matrix is consistent, the value of CI is 0. The larger the value of CI, the worse the consistent performance of the matrix.

*(3) The Corresponding Random Consistency Index RI Mean Value Needs to Be Found*. The RI value is the average of the random consistency index. Experts construct 100 samples by random sampling. Random sampling from 1 to 10 is required. Its inverse numerical construction is a reciprocal matrix. The largest eigenroot for which the mean value of *λ*_max_ needs to be calculated.

(4) $$\begin{array}{c} \text{RI}=\frac{\lambda_{\max}^{\prime }-n}{n-1}. \end{array}$$

*(4) The Matrix Consistency Coefficient CR Needs to Be Calculated*. When the number of layers is less than or equal to 2, the matrix will maximize close to complete consistency. When the number of layers is greater than 2, the consistency coefficient CR is the random consistency ratio of the matrix.

(5) $$\begin{array}{c} \text{CR}=\frac{\text{CI}}{\text{RI}}. \end{array}$$

According to each secondary influencing factor, the weight value and the consistency ratio are calculated in the established judgment matrix. The judgment matrix, weight, and CR value of each index are shown below.

(6) $$\begin{array}{c} A=\left[\begin{array}{ccccc} 1 & 1/2 & 1/3 & 1 & 1/4\\ 2 & 1 & 1/2 & 2 & 1/3\\ 3 & 2 & 1 & 3 & 1/2\\ 1 & 1/2 & 1/3 & 1 & 1/4\\ 4 & 3 & 2 & 4 & 1 \end{array}\right]. \end{array}$$

After calculating the weight value of each first-level index, it is shown in Figure 8.

After calculation, the maximum eigenvalue is 5.073. CI = 0.016, RI = 1.02, and CR = 0.014. When CR is less than 0.1, the consistency of the judgment matrix is considered acceptable.

The judgment matrix, weight, and CR value statistical results of *a*~*e* sub-indices are as follows.

(7) $$\begin{array}{c} A_{1}=\left[\begin{array}{cc} 1 & 1/2\\ 1/2 & 1 \end{array}\right], \end{array}$$

(8) $$\begin{array}{c} A_{2}=\left[\begin{array}{cccc} 1 & 1/3 & 1/4 & 1/2\\ 3 & 1 & 1/2 & 2\\ 4 & 2 & 1 & 2\\ 2 & 1/2 & 1/2 & 1 \end{array}\right], \end{array}$$

(9) $$\begin{array}{c} A_{3}=\left[\begin{array}{ccccc} 1 & 4 & 3 & 2 & 2\\ 1/4 & 1 & 1/2 & 1/2 & 1/3\\ 1/3 & 2 & 1 & 1 & 1\\ 1/2 & 2 & 2 & 2 & 1/2\\ 1/2 & 3 & 1 & 1 & 1 \end{array}\right], \end{array}$$

(10) $$\begin{array}{c} A_{4}=\left[\begin{array}{cc} 1 & 1\\ 1 & 1 \end{array}\right], \end{array}$$

(11) $$\begin{array}{c} A_{5}=\left[\begin{array}{cccc} 1 & 1/3 & 1/5 & 1/5\\ 3 & 1 & 1/2 & 1/2\\ 5 & 2 & 1 & 1\\ 5 & 2 & 1 & 1 \end{array}\right]. \end{array}$$

After calculating the weight value of each second-level indicators, it is shown in Figure 9.

After calculation, the maximum *A*_1_ eigenvalue is 2.00. CI = 0.00, RI = 0.01, and CR = 0.00. When CR is less than 0.1, the consistency of the judgment matrix is considered acceptable. After calculation, the maximum *A*_2_ eigenvalue is 4.18. CI = 0.06, RI = 0.80, and CR = 0.08. When CR is less than 0.1, the consistency of the judgment matrix is considered acceptable. After calculation, the maximum *A*_3_ eigenvalue is 5.033. CI = 0.008, RI = 1.02, and CR = 0.008. When CR is less than 0.1, the consistency of the judgment matrix is considered acceptable. After calculation, the maximum *A*_4_ eigenvalue is 2.00. CI = 0.00, RI = 0.01, and CR = 0.00. When CR is less than 0.1, the consistency of the judgment matrix is considered acceptable. After calculation, the maximum *A*_5_ eigenvalue is 4.15. CI = 0.05, RI = 0.80, and CR = 0.06. When CR is less than 0.1, the consistency of the judgment matrix is considered acceptable.

### 6.4. Fuzzy Comprehensive Evaluation Method

The evaluation of the project is a fuzzy evaluation method. Three field engineers with qualifications in technical construction management and two experts in construction, environmental protection, and other fields are invited to form an evaluation team. The five members will rate the green construction of the project around the content of the aforementioned 17 factors. The specific index scoring results are shown in Figure 10.

According to the weight value and score value of each index, the fuzzy comprehensive evaluation result of each level is calculated.

1. It is necessary to calculate the fuzzy comprehensive evaluation set and index score of *a* factor.

(12) $$\begin{array}{c} \left\{\begin{array}{c} B_{a}={WR}_{a}=\left(\begin{array}{cc} 0.9 & \begin{array}{cc} 0.1 & \begin{array}{cc} 0 & 0 \end{array} \end{array} \end{array}\right)\\ S_{a}=\left(\begin{array}{c} \begin{array}{ccc} 0.9 & 0.1 & 0 \end{array} \end{array}\right)\times \left(\begin{array}{c} \begin{array}{cc} 100 & \begin{array}{cc} 80 & \begin{array}{cc} 60 & 0 \end{array} \end{array} \end{array} \end{array}\right)=98 \end{array}\right.. \end{array}$$

(2) It is necessary to calculate the fuzzy comprehensive evaluation set and index score of *b* factor.

(13) $$\begin{array}{c} \left\{\begin{array}{c} B_{b}={WR}_{b}=\left(\begin{array}{c} \begin{array}{cc} 0.372 & \begin{array}{cc} 0.394 & \begin{array}{cc} 0.234 & 0 \end{array} \end{array} \end{array} \end{array}\right)\\ S_{b}=\left(\begin{array}{c} \begin{array}{cc} 0.372 & \begin{array}{cc} 0.394 & \begin{array}{cc} 0.234 & 0 \end{array} \end{array} \end{array} \end{array}\right)\times \left(\begin{array}{c} \begin{array}{cc} 100 & \begin{array}{cc} 80 & \begin{array}{cc} 60 & 0 \end{array} \end{array} \end{array} \end{array}\right)=82.76 \end{array}\right.. \end{array}$$

(3) It is necessary to calculate the fuzzy comprehensive evaluation set and index score of *c* factor.

(14) $$\begin{array}{c} \left\{\begin{array}{c} B_{c}={WR}_{c}=\left(\begin{array}{c} \begin{array}{cc} 0.596 & \begin{array}{cc} 0.404 & \begin{array}{cc} 0 & 0 \end{array} \end{array} \end{array} \end{array}\right)\\ S_{c}=\left(\begin{array}{c} \begin{array}{cc} 0.596 & \begin{array}{cc} 0.404 & \begin{array}{cc} 0 & 0 \end{array} \end{array} \end{array} \end{array}\right)\times \left(\begin{array}{c} \begin{array}{cc} 100 & \begin{array}{cc} 80 & \begin{array}{cc} 60 & 0 \end{array} \end{array} \end{array} \end{array}\right)=91.92 \end{array}\right.. \end{array}$$

(4) It is necessary to calculate the fuzzy comprehensive evaluation set and index score of *d* factor.

(15) $$\begin{array}{c} \left\{\begin{array}{c} B_{d}={WR}_{d}=\left(\begin{array}{c} \begin{array}{cc} 0.7 & \begin{array}{cc} 0.3 & \begin{array}{cc} 0 & 0 \end{array} \end{array} \end{array} \end{array}\right)\\ S_{d}=\left(\begin{array}{c} \begin{array}{cc} 0.7 & \begin{array}{cc} 0.3 & \begin{array}{cc} 0 & 0 \end{array} \end{array} \end{array} \end{array}\right)\times \left(\begin{array}{c} \begin{array}{cc} 100 & \begin{array}{cc} 80 & \begin{array}{cc} 60 & 0 \end{array} \end{array} \end{array} \end{array}\right)=94 \end{array}\right.. \end{array}$$

(5) It is necessary to calculate the fuzzy comprehensive evaluation set and index score of *e* factor.

(16) $$\begin{array}{c} \left\{\begin{array}{c} B_{e}={WR}_{e}=\left(\begin{array}{c} \begin{array}{cc} 0.478 & \begin{array}{cc} 0.522 & \begin{array}{cc} 0 & 0 \end{array} \end{array} \end{array} \end{array}\right)\\ S_{e}=\left(\begin{array}{c} \begin{array}{cc} 0.478 & \begin{array}{cc} 0.522 & \begin{array}{cc} 0 & 0 \end{array} \end{array} \end{array} \end{array}\right)\times \left(\begin{array}{c} \begin{array}{cc} 100 & \begin{array}{cc} 80 & \begin{array}{cc} 60 & 0 \end{array} \end{array} \end{array} \end{array}\right)=89.56 \end{array}\right.. \end{array}$$

The final fuzzy comprehensive evaluation set and comprehensive evaluation scores are calculated as follows.

(17) $$\begin{array}{c} \left\{\begin{array}{c} B=WR=\left(\begin{array}{c} \begin{array}{cc} 0.551 & \begin{array}{cc} 0.414 & \begin{array}{cc} 0.035 & 0 \end{array} \end{array} \end{array} \end{array}\right)\\ S=\left(\begin{array}{c} \begin{array}{cc} 0.551 & \begin{array}{cc} 0.414 & \begin{array}{cc} 0.035 & 0 \end{array} \end{array} \end{array} \end{array}\right)\times \left(\begin{array}{c} \begin{array}{cc} 100 & \begin{array}{cc} 80 & \begin{array}{cc} 60 & 0 \end{array} \end{array} \end{array} \end{array}\right)=90.32 \end{array}\right.. \end{array}$$

According to the principle of maximum membership degree in fuzzy mathematical theory, in this case, the green evaluation of the project is good within the range. At the same time, the overall evaluation score of 90.32 is that green buildings are better projects.

## 7. Related Suggestions

Based on the evaluation results of this project, relevant suggestions are put forward as follows.

### 7.1. Strengthen the Green Construction Concept of Sustainable Development

The World Commission on Environment and Development points out that there are many legal issues that need to be addressed urgently. Administrative and economic measures cannot solve all the problems caused by pollution. It is also one of the main reasons for the failure to overcome further environmental decline. Most people in the world have not adapted to the new environment of science and technology in modern industrial society. The masses in China know very little about green buildings, and people's understanding of green buildings is not enough. This has influenced the wider promotion of green buildings. By raising awareness of the advanced concepts of green building, all employees should strengthen publicity and education awareness and strengthen construction workers to carry out green building, green building inspection, and inspection activities. Initiative and self-awareness must be increased. The standard construction company needs to be handed over to the unqualified construction company within the rectification period.

### 7.2. Focus on Policy Guidance and Incentives for Green Construction

The construction sector should learn lessons from the successful practices of advanced countries and speed up the formulation of regulations. In turn, green construction can be promoted, and policies, laws, and regulations can be established and improved as soon as possible. According to the requirements of construction enterprises, relevant departments shall carry out green construction in accordance with regulations. Financial, taxation, and other economic means can be used to establish an effective incentive mechanism and enhance the enthusiasm and initiative of enterprises to independently implement green construction. The construction of construction projects in the green construction evaluation process needs to meet the standards of tax reduction for construction companies and offset the increased costs of green construction measures. It is necessary to meet the standard of raising tax rates for construction companies and increase the cost of social responsibility. A system conducive to promoting green construction should be established. The construction drawings and environmental technical requirements that encourage green construction, such as construction contract responsibilities, are complied with by contractors during construction supervision. It is necessary to improve green building management methods, make green buildings more colorful, and create a good environment. It is a civilized construction management measure.

### 7.3. Build a Reasonable and Effective Green Construction Technology System

Green building construction technology is the main research object. It is necessary to start from the construction technology, find out the construction production law and master the production construction characteristics. It can analyze the construction production factors and the construction technology of some reconstruction projects. By studying the particularity of construction and production, green construction can be effectively promoted. Green building technology research has established positive results and useful experience in environmental engineering technology. There is a need to learn lessons from experience and guide green construction.

### 7.4. Improve the Green Construction Management System

According to the design documents for environmental protection and construction bidding documents, clarify the requirements of the construction unit responsible for the environmental responsibility in the contract. The construction unit in the construction phase of the construction project shall strictly abide by the environmental laws, regulations, policies, and measures for environmental protection, pollution prevention, and ecological protection in the engineering design documents. The designated representative designated by the owner and the project manager designated by the construction unit are directly responsible for the green construction site. The owner and the construction unit shall establish a construction site environmental management system and personnel responsibilities. It consists of project managers, to build environmentally friendly network operators. The owner and the construction unit shall actively adopt the IS014000 environmental management system and the IS09001 quality management system. Such activities are carefully carried out by perfecting the project construction, environmental protection, and green construction standards, and setting standards for the environmental management system.

## 8. Conclusion

With the rapid development of China's economy, the people have higher and higher requirements for the quality of life, and the development of green buildings in China is very fast. Many developers are not aware of this and lack effective management experience. This has led to various problems in the cost control of green building projects. BIM can not only comprehensively sort out and update complex commercial project information, but also provide an information platform for mutual communication between different stages and different participants in the entire life cycle of a construction project. By promoting the effective flow of information among all parties, it can improve the competitiveness of enterprises and enhance the cost control ability of enterprises.

Green building is the development trend of the future construction industry. As a building information model, BIM is also an inevitable direction for the development of information in the construction industry. Green BIM is the focus of the future development of the construction industry. Therefore, the research on the application mechanism of BIM in green building project management is an important guarantee for the application of BIM in green buildings. The establishment of BIM model in green building project management for comprehensive evaluation is an important research content. By constructing an evaluation model for the application of BIM technology in green building project management, the problems that arise in the application of BIM technology in green buildings are reflected. The corresponding work can be adjusted in time to help the effective management of green building projects and the promotion and improvement of BIM technology.

## Figures and Tables

**Figure 1:** The change law of the total output value and the number of construction companies applying BIM in the construction industry in the past ten years.

**Figure 2:** Status quo of informatization application in construction industry.

**Figure 3:** Changes brought by BIM in engineering construction.

**Figure 4:** The proportion of major accidents caused by construction project management level in the past ten years.

**Figure 5:** The proportion of structured and unstructured building information to green building information.

**Figure 6:** Project participants in the green building implementation process.

**Figure 7:** The complete model framework constructed.

**Figure 8:** Weight value of first-level indicators.

**Figure 9:** Weight value of second-level indicators.

**Figure 10:** The specific index scoring results. (a) index score. (b) Index score. (c) Index score. (d) Index score.

## Data Availability

The data used to support the findings of this study are available from the corresponding author upon request.
